# Dry Ice in Decoverslipping Microscopic Slides: A Novel Approach

**DOI:** 10.7759/cureus.103947

**Published:** 2026-02-20

**Authors:** Soujanya Pinisetti, Alivelu Dasarathi, M Jyothsna, Heera Shaik, Jomyir Jini, Rizwana Iqbal

**Affiliations:** 1 Department of Oral Pathology, Government Dental College and Hospital, Kadapa, IND; 2 Department of Oral and Maxillofacial Pathology, Government Dental College and Hospital, Kadapa, IND

**Keywords:** decoverslipping, dry ice, histopathological slides, restaining, xylene

## Abstract

Introduction: Histopathological slides play a pivotal role in diagnostic pathology; however, over time, preserved slides may exhibit fading of staining quality, thereby diminishing their diagnostic and research value. Histopathological laboratories perform coverslip removal techniques to enable restaining of histopathological slides. Conventionally, xylene is used for coverslip removal; however, it is a time-consuming process. To tackle this, dry ice, a widely accessible and cost-effective cooling agent with a low freezing point (-78.5°C), was used for coverslip removal and compared with conventional xylene.

Aim: This study aimed to evaluate the effectiveness of dry ice vs xylene in decoverslipping microscopic slides.

Materials and methods: A retrospective study was conducted by the Department of Oral and Maxillofacial Pathology and Microbiology, in which 56 archival slides collected over a 15-year period were randomly selected for coverslip removal. These faded slides were categorized into four groups, each denoting a four-year interval, and evenly divided between dry ice and xylene. Coverslip removal time was recorded with a stopwatch, and slides were examined under a stereomicroscope for tissue damage and then immersed in xylene to eliminate residual dibutylphthalate polystyrene xylene (DPX). Finally, tissue sections were restained with hematoxylin and eosin (H&E) stain.

Result: The mean time required for coverslip removal with dry ice was 65 ± 17.760 seconds, whereas xylene required 4 ± 1.440 days. Dry ice caused minor tissue distortion, though not statistically significant (p = 0.075). After H&E restaining, both procedures produced comparable staining results (p = 1.00).

Conclusion: Dry ice removes coverslips quicker and more effectively than xylene, with minimal tissue distortion and preserved staining quality. It also avoids xylene's adverse health and environmental effects, making it an improved laboratory choice.

## Introduction

Microscopic slides used in histopathology serve as essential tools for diagnosing and fulfilling long-term needs such as research, education, and retrospective case reviews [1].Tissue sections are placed on microscopic slides using a coverslip and dibutylphthalate polystyrene xylene (DPX) mounting media to preserve the stained section. However, prolonged contact with the mounting medium can cause these microscopic slides to fade or get discolored over time [2]. When the original tissue block is not accessible for re-sectioning, histopathology labs often need to decoverslip and restain these archived slides in order to restore their diagnostic quality [1].

Traditionally, xylene has been used for decoverslipping, but it is a time-consuming process ranging from a few hours to several days. Xylene exposure also poses significant toxic and occupational hazards, affecting various organ systems and causing side effects that may begin as dizziness, nausea, and headaches, to more serious systemic toxicity. These health risks highlight the significance of avoiding xylene exposure, especially in laboratory and industrial settings [3].

To minimize the hazardous effects of xylene and the time-consuming process of decoverslipping, it was essential to develop a rapid process for removing coverslips. As alternatives to the conventional xylene immersion technique, approaches involving liquid nitrogen, ultrasonic vibration, and freezing temperatures were explored in the past to accelerate the decoverslipping process, but none showed promising results. However, among them, liquid nitrogen showed considerable effectiveness but had certain limitations [1].

Dry ice is the solid form of carbon dioxide, with its extremely low freezing point (-78.5°C), which enables rapid and efficient cooling. It is inexpensive, widely available, and extensively used across the medical, pharmaceutical, and food industries, as well as in laboratories for the refrigeration, storage, and transportation of vaccines and medical supplies. Considering its physicochemical properties, notably its low sublimation temperature and established use across various applications, dry ice was considered a potential candidate for evaluation as a decoverslipping agent. To the best of our knowledge, only a few studies have been reported in the literature. Therefore, the present study aimed to assess the effectiveness of dry ice in removing coverslips from histopathology slides as a possible alternative to conventional xylene-based methods.

## Materials and methods

A total of 56 archived hematoxylin and eosin (H&E)-stained histopathological slides (n = 56), prepared over the past 15 years and exhibiting signs of fading, were uniformly mounted with DPX as the mounting media and retrieved from the institution's archives. These archived slides were chosen to compare the effectiveness of two different coverslip removal techniques: the dry ice method and the conventional xylene method. The slides were categorized into four groups: group 1 comprised 14 slides taken from 2008 to 2011 (n = 14), group 2 comprised 14 slides taken from 2012 to 2015 (n = 14), group 3 comprised 14 slides taken from 2016 to 2019 (n = 14), and group 4 comprised 14 slides taken from 2020 to 2023 (n = 14). Each group was further divided into two subgroups based on the method chosen: subgroup A (coverslips removed using the dry ice method) and subgroup B (coverslips removed using the conventional xylene method).

Decoverslipping of the faded microscopic slides was carried out in a well-ventilated area of the histopathology lab at the Government Dental College and Hospital in Kadapa, India, after obtaining approval from the institute's Institutional Ethics Committee (approval number: Pr.43/IEC/GDCH/2025-26). Dry ice (-78°C) used during the procedure was temporarily stored in a thermal ice pack container. Each faded microscopic slide was assigned a unique identifying number. Faded microscopic slides were mounted with coverslips, and the surface bearing the coverslip was carefully placed on dry ice at -78.5°C (Figure 1). Due to the extremely low temperature, handling was done using protective gloves, and a stopwatch was set to monitor the exposure time [2].

**Figure 1:** Placement of microscopic slides on dry ice

At the designated time point, the microscopic slides were taken off the dry ice, and the coverslips were gently raised using an old microtome blade (Figure 2). The coverslips were expected to detach effortlessly from the slide surface without requiring any additional force from the operator. If any difficulty is encountered while lifting the coverslip, the faded microscopic slide should be returned to the dry ice for a few additional seconds. After this brief re-exposure, the same removal technique is reapplied.

**Figure 2:** Coverslip removal using disposable microtome blade after 45 seconds

Following coverslip removal, residual DPX mountant often remains on the faded microscopic slides (Figure 3). This remnant can be eliminated by immersing the slides in xylene for five minutes (Figure 4, Figure 5). In subgroup B, faded slides are directly immersed in xylene contained within Coplin jars. As per conventional practice, xylene typically requires several days to a week for the coverslip to loosen and settle at the bottom of the Coplin jars.

**Figure 3:** Residual mounting media left on the slide after coverslip removal

**Figure 4:** Removal of DPX by the placement of coverslip dislodged slides inside a Coplin jar with xylene DPX: dibutylphthalate polystyrene xylene

**Figure 5:** Air-drying the slides after coverslip removal

Subsequently, the slides were examined under a stereomicroscope to assess any potential tissue distortion. After coverslip removal, the microscopic slides are restained with H&E to evaluate any tissue loss or alterations in morphological changes (Figure 6, Figure 7). The stained slides were evaluated by four independent observers using the following grading system: good indicates equal or superior staining intensity, fair indicates a lower intensity, and "poor" signifies inadequate staining intensity or a lack thereof.

**Figure 6:** Archival slide with faded H&E stain H&E: hematoxylin and eosin

**Figure 7:** Restained after decoverslipping

## Results

Table 1 shows that the mean time required for coverslip removal using dry ice was 65 ± 17.760 seconds and the mean time required for coverslip removal using xylene was 4 ± 1.440 days.

**Table 1:** Macroscopic parameter: mean time taken for the removal of coverslip

Agent used for coverslip removal	Mean time	Standard deviation
Dry ice	65 seconds	17.760
Xylene	4 days	1.440

Table 2 shows tissue distortion with dry ice, whereas all xylene-treated slides remained intact. The p-value was 0.75 (p < 0.05) indicating no significant difference between the two agents.

**Table 2:** Macroscopic parameter: distortion of tissue section after coverslip removal Chi-squared test (p < 0.05)

Agent used for coverslip removal	Distortion of tissue		Total	P-value
	Yes	No		
Dry ice	3	25	28	0.75
Xylene	0	28	28	

Table 3 shows that both xylene and dry ice showed comparable results, with most sections exhibiting good staining and a few showing poor quality. A chi-squared value of 1.000 (p > 0.05) indicated no significant difference between the two coverslip removal agents.

**Table 3:** Quality of stain after coverslip removal from the faded microscopic slides Chi-squared test (p < 0.05)

Agent used for coverslip removal	Staining			Total	P-value
	Good	Fair	Poor		
Dry ice	16	11	1	28	1.000
Xylene	16	11	1	28	

When microscopic slides were placed on dry ice with the coverslip facing downward for more than a couple of minutes, the entire tissue section tended to detach along with the coverslip. Therefore, during coverslip removal, it was necessary to monitor the loosening of the coverslip at 20-second intervals to prevent complete tissue loss or distortion.

## Discussion

Histopathological slides are often preserved for research purposes and serve as valuable resources in undergraduate and postgraduate education. Over time, these slides often show fading of stains due to aging and mountant, which can compromise their diagnostic and teaching utility. When the original tissue block is not available, removing the coverslip and restaining the section become essential to restore staining quality and diagnostic clarity [1,2].

Coverslip removal is often required in several applications, including molecular research for DNA extraction, investigations into targeted therapies, preparation of neuronal cultures, and diagnostic evaluation of conditions such as lung adenocarcinoma, soft tissue neoplasms, and thyroid pathologies [2,4].Conventionally, xylene has been used for coverslip removal; however, it has certain limitations like being time-consuming and having toxic effects. Hence, other alternative methods have been employed for removing coverslips like liquid nitrogen, freezing temperature, and ultrasonic vibration.

Zhou et al. implemented liquid nitrogen for coverslip removal to facilitate DNA and RNA extraction and integrity [5].However, Cozma and Henwood highlighted that there are slide fracturing and tissue detachment, emphasizing that although nucleic acid preservation is achieved, maintaining tissue architecture is critical for reliable microscopic analysis. Another approach employed by Cozma and Henwood was freezing temperature (-80°C), in which freezing the mountant media beneath the coverslip led to its cracking, making its handling in regular running laboratories difficult [1]. Rainbow's ultrasonic vibration approach causes significant tissue loss after the coverslip loosening; it also requires constant supervision by skilled technicians, making it unsuitable for use in busy laboratories with limited manpower [6].Pedraza and Marciano described a humidity-based method for coverslip removal using nail polish to prevent cracking. While effective, it requires multi-day incubation and may cause minor cracks if the polish is inadequate or the coverslip isn't fully loosened, sometimes requiring retreatment [7].

The present comparative study evaluated dry ice and xylene methods for removing coverslips from DPX-mounted slides aged between 2008 and 2023. The results demonstrated that dry ice successfully removed coverslips within a mean time of 65 seconds compared to xylene, which took a mean time of four days for coverslip removal, irrespective of slides aged between one and 15 years. A faster coverslip removal technique involved applying dry ice (solid CO₂ at 78.5°C) to the slides, which froze the DPX mounting medium, immobilizing its molecular chains. The subsequent thermal contraction created micro-fissures at the DPX-glass interface due to differential shrinkage, weakening the adhesive bond and allowing the coverslip to be lifted off easily within a few seconds. Importantly, this method induces no chemical alteration in the DPX relying solely on physical changes from rapid cooling.

Coverslip removal using the conventional xylene method typically requires several days and may extend up to a week. Due to prolonged immersion (several hours to days) in xylene, an aromatic hydrocarbon dissolves the resin-based DPX mounting media, allowing gentle coverslip removal without mechanical force and preserving the underlying tissue section.

Following coverslip removal, stereomicroscopic examination revealed tissue distortion in three slides processed with the dry ice method. The distortion was attributed to overexposure exceeding two minutes, which can dehydrate the tissue and render it brittle, increasing the susceptibility to tissue fragmentation during coverslip removal. The distortion was statistically insignificant (p > 0.05) and did not compromise diagnostic quality, while xylene-treated slides exhibited no tissue distortion because xylene is a non-polar organic solvent. This means it doesn’t interact with water-based tissue components; rather, instead of tissue, it dissolves the mounting medium (resin-based DPX) without affecting the underlying tissue, allowing the coverslip to detach gently.

After restaining, four independent observers graded the staining quality as good, fair, or poor, with no significant differences between dry ice and xylene groups (p = 1.000). Dry ice, used for rapid freezing, does not chemically alter proteins or nucleic acids, preserving stainable tissue components; xylene, as a clearing agent, removes wax and dissolves mounting media without interacting with tissue proteins or dyes. Both dry ice and xylene do not disrupt staining quality when used appropriately, as they preserve tissue integrity and do not chemically interfere with stainable components.

Various methods for coverslip removal were mentioned in the literature with certain limitations like being time-consuming, causing tissue distortion, being technique-sensitive and expensive, requiring special handling, and necessitating safety precautions. However, in this study, the results support the use of dry ice as a rapid and efficient method for restoring faded microscopic slides while maintaining tissue morphology, avoiding cracks in the microscopic slides, and preserving staining quality compared to the traditional xylene method.

## Conclusions

Archived histological slides often exhibit diminished staining clarity over time, rendering them unsuitable for diagnosis. To restore their diagnostic utility, restaining is necessary, which requires the removal of the coverslip, which is commonly done with xylene and might take several days or weeks. In comparison, the present study evaluates the use of dry ice as a rapid and efficient alternative, achieving coverslip detachment within approximately 65 seconds. Notably, the dry ice method preserved tissue integrity and staining integrity while eliminating the health and environmental hazards associated with xylene exposure. The comparative analysis demonstrated that dry ice offers a significantly faster and safer approach to coverslip removal, with the superior preservation of histological quality.
